# The role of the arts on community mental health and cultural understanding in Addis Ababa, Ethiopia

**DOI:** 10.3389/fpubh.2023.1253645

**Published:** 2023-11-17

**Authors:** Mary O. Hearst, Melaku Belay, Hui Wilcox

**Affiliations:** ^1^Child and Family Health, University of Minnesota Twin Cities, St. Paul, MN, United States; ^2^Fendika Cultural Center, Addis Ababa, Ethiopia; ^3^Kofi Annan Institute for Global Citizenship, St. Catherine University, Saint Paul, MN, United States

**Keywords:** Ethiopia, mental health, culture, art, social cohesion

## Abstract

**Background:**

In low-and middle-income countries, there are rising rates of depression and anxiety. In Ethiopia, depression and anxiety rates were rising before the COVID-19 pandemic, and the country faces ethnic discord and armed conflict. Novel community-based strategies are needed to improve mental health and cultural unity. The purpose of this research was to describe the role of a cultural center’s art programming in mental health and cultural unity.

**Methods:**

This qualitative study conducted interviews and focus groups with audience members, artists, and staff at Fendika Cultural Center, Addis Ababa, in January 2023. Participants were recruited via word of mouth and purposive sampling. Focus groups and interviews led in English or Amharic were recorded, transcribed, and translated as needed. Questions included participant experiences with Fendika Cultural Center and how experiencing the arts at Fendika influences wellbeing. We used deductive analysis, guided by the Arts and Culture in Public Health Framework.

**Results:**

Two focus groups (*n* = 11 participants, five females and six males) and five key informant interviews (three females and two males) were completed. Findings suggested that the activities at Fendika were important for addressing individual depression and anxiety through the social and physical environments as well as the inherent cultural support and unity expressed through the arts. The themes were consistent with the Arts and Culture in Public Health Framework.

**Conclusion:**

The arts play an important role in positive mental health and cultural unity. Further research is needed to establish the generalizability, reach, and persistence of the impact of cultural centers on mental health cultural understanding.

## Background

The past decade has seen a dramatic rise in anxiety and depression globally. Since 2017, there has been a 13% increase in mental health conditions globally and poor mental health afflicts one in five persons from post-conflict situations (1). The World Health Organization estimates that costs associated with depression and anxiety alone exceed $1 trillion US dollars (USD) (1). Disability-adjusted life years (DALYs) for depression and anxiety were 577.7 and 360.1 per 100,000 globally and 605.9 and 315.9 for low-and middle-income countries, respectively (2). A recent meta-analysis shows that the rates of anxiety and depression were higher across the African continent than in other regions. Although the data were incomplete (3), the rise in anxiety and depression widened the already large treatment gap in mental health services across low-and middle-income countries (4). Ethiopia, the second most populated country in Africa (5), is an example of a country experiencing a generalized rise in mental health disorders and elevated levels of depression and anxiety pre-COVID-19 pandemic. In Ethiopia specifically, DALYs for depression were 808.7 per 100,000 and 339.1 per 100,000 for anxiety in 2019 (2).

Specific attention to Ethiopia is notable because, including the COVID-19 pandemic (6), the country faced an armed conflict in the Tigray region from November 2020 to November 2021, although clashes continued in 2023, resulting in unprecedented internal displacement, violence, cruelty, and furthering the mental health crisis (7–10). Additionally, Ethiopia has a long history of internal conflict between ethnic groups. There are 100 languages spoken in Ethiopia, although Amharic and Oromo are the most common (5). There are many reasons for the ongoing conflict, including, but not limited to, uncertainty and instability, historical memories of grievances, and systematic intolerance (11). From 1991 to 2012, the Tigray People’s Liberation Front (TPLF) dominated national leadership, ruled as an autocracy, and marginalized the majority Somali, Oromo, and Amhara ethnic groups until the death of the soldier-politician Meles Zenawi. The TPLF continued to govern Ethiopia until 2018, when Prime Minister Abiy Ahmed Ali, who is ethnically Oromo, became prime minister (7, 11). Ethnic conflict and violence continue in Ethiopia to this day (7, 12–14). In early 2023, a split in the Orthodox Church resulted in violent riots between ethnic groups in Addis Ababa and a government shutdown of social media (15). The country faces extreme internal pressure and division, magnified by political pundits.

Given the rising burden of poor mental health coupled with inadequate health services, a broader and more comprehensive approach is needed to address the multifaceted aspects of life in Ethiopia and elsewhere. In rebuilding the health systems of care, further engagement at the community level and building social support networks also play an important role (4, 16). The global public health movement needs to embrace cross-sectoral and interdisciplinary partnerships to address the increasingly complex and seemingly intractable needs of communities. The systemic issues exacerbating mental health crises, such as armed conflict, global pandemics, and a lack of cross-cultural acceptance, cannot be solved by traditional science alone. One relatively novel public health approach is intervention through the arts.

The role of the arts, including music, dance, and creative expression, as a mechanism for community health is relatively new to the field of public health; however, art as a therapeutic modality has been used as a means of healing and improving individual health for centuries (17). The bonds of culture unite people (18), and cultural expression and cross-cultural appreciation can be manifested through the arts. The arts can also be used as a tool for expressing complex emotions and as a form of communication to increase understanding of the social and structural conditions underlying health equity (19). Moreover, the arts can be used to mitigate the impact of social and structural factors that interfere with health equity (20). Finally, the arts as a form of health communication can empower communities and engage people emotionally in the health topic (21).

Addis Ababa is the capital city of Ethiopia and is the location of the Fendika Cultural Center, a venue in which there is cross-cultural music, dance, visual art, and an open gathering place. Fendika Cultural Center (herein Fendika) is a cultural oasis and unique revitalized space in Addis Ababa^1^ that historically housed Azmari music and dancers. The mission of Fendika is to celebrate and renew Ethiopia’s rich cultural heritage, seeking peace, and humanity’s unity (22). The purpose of this qualitative study was to explore the ways in which art—delivered through a cultural center—can impact mental health, build social support, and create cultural unity for the artists who perform, the staff, the audience members, and public health professionals. This research provides a further understanding of culturally specific contexts and processes in which healing takes place through the arts.

## Methods

### Study location

This qualitative study was conducted in January 2023 at Fendika. Fendika was established in 2016, although the venue opened in the early 1990s as an Azmari Bet, or a house of Azmaris, who are traditional musicians who improvise singing directly to audiences. Melaku Belay, the owner of Fendika since 2016, has a deep belief in the power of the arts in building communities that have been infused into the center. The space has continued to grow and offers live music and dance programs, an art gallery, and family arts programming.

### Participants

Participants were drawn from four distinct sources using purposive sampling. Artists and Fendika staff were approached by the study team to determine their interest and availability to participate. Artists were those who performed, presented, or curated the arts at the center. Audience members were identified by the study team while visiting Fendika events through word of mouth and invitations directed at casual acquaintances known to attend Fendika events. Potential participants were told about the purpose of the study, and if interested, an interview was arranged. One public health leader was purposefully invited, given her former role with the World Health Organization, being Ethiopian, and currently working on public health initiatives in Ethiopia.

### Framework: arts and culture in public health framework

*A priori* analysis, the Arts and Culture in Public Health Framework was identified as the analytic framework because it aligned with the study’s aim to explore the arts related to mental health, social support, and cultural unity (21). The evidence-based framework was designed using the social ecological framework and extensive community and organizational stakeholder input (21). The framework provides a roadmap of the evidence-based links between exposure to the arts, participation in the arts, and health outcomes. The framework identifies seven mechanisms by which six-health outcome areas are achieved (Figure 1). In line with the primary purpose of the study, the outcomes and related mechanisms chosen were: (1) providing direct health benefits, including stress reduction, increased social cohesion, and reduced loneliness, and increased happiness and wellbeing; (2) creating safe, inclusive, and engaging environments, including cultural and historical representation, civic pride, and engagement; and (3) supporting social, cultural, and policy change, including enabling dialogue within or across groups, increasing social cohesion, elevating underrepresented voices, and increasing community capacity and resilience; and although secondarily (21).

**Figure 1:** Framework for Arts and Culture in Public Health: an evidence-based framework. Taken from Sonke and Golden (21).

### Qualitative data collection

Prior to the initiation of focus groups or interviews, participants completed the informed consent process in English or Amharic. All focus groups and interviews had extensive notes taken, recorded, and transcribed, if in Amharic. The focus group and interview questions included similar core questions with prompts and follow-up questions (Table 1). Participants shared their first name, how they interface with Fendika (staff, artist, or audience member), how often they attend Fendika, and what type of event they typically attend. Participants were identified as male or female only. No other demographic data were collected. The public health official was asked questions more generally about the role of the arts, such as: (1) Do you think the arts have a role in community health? How and why, or why not? (2) Do you think the arts can help unite cultures? How and why, or why not? and (3) How do the Ministry of Health and the public health community use art to improve health? The Institutional Review Board of REDACTED approved this study and declared it exempt.

**Table 1:** Core and examples of supplementary questions asked of participants in focus groups and interviews of artists, staff, and audience members, Addis Ababa, Ethiopia 2023.

Core questions “Fendika” represents the arts including music, dance, art gallery, and family art day	Supplementary questions
Introduction: name and role	What do you mean by (e.g., “healing”)? Provide examples
How often do you attend Fendika?	Why do you think some people feel it is inappropriate to go there?
What events do you typically attend?	How did you cope?
What is your Fendika experience? Or What do you get out of Fendika?	Inspiring, in what ways?
How do you describe the Fendika essence/vibe/mood?	How has Fendika influenced you as a person today?
Do you see that Fendika has any role in the larger society?	
How did you get to know Fendika?	
Does Fendika impact health? In what ways?	
Have you observed a broader impact of Fendika? For example, related to the war/COVID-19.	
How has the war or ethnic conflict been at Fendika?	

Participants shared their first name, how they interface with Fendika (staff, artist, or audience member), how often they attend Fendika, and what type of event they typically attend.

### Analysis

A deductive approach was determined *a priori* using the Arts and Culture in Public Health Framework (21) as the themes and identifying excerpts that fit the codes (23). Notes and transcripts were reviewed by two researchers; one researcher identified the excerpts and assigned a thematic code, and the second researcher validated the coding. Written notes were transcribed and reviewed with the transcripts in a word-processing document. The themes were organized in a spreadsheet. The word-processing document was used to identify excerpts, which were copied into the spreadsheet. The spreadsheet organized the data, including attribute codes (interview vs. focus group, participant sex, and the participant’s role), thematic area, and transcript excerpts representing the thematic area (24). Qualitative software was not used for simplicity, transferability with team partners, or the determination that the qualitative software advantage of organizing, not analyzing, data had no additional benefits for this analysis (25). The final stage was to examine the thematic areas and designate excerpts into a mechanism from the evidence-based framework. Following analysis, a fourth thematic area was added to the framework, which included (4) increasing health service equity and access, including increased access and engagement, facilitating dialogue even about difficult issues across differences, and delivering services in a more culturally responsive manner.

### Results

Two focus groups and five individual interviews were completed. Participants included eight men (six from focus groups and two from individual interviews) and eight women (five from focus groups and three from individual interviews). The results are organized into the four thematic areas based on the study purpose and the Arts and Culture in Public Health Framework (21): (1) direct health benefits; (2) safe, inclusive, and engaging environment; (3) social, cultural, and policy change; and (4) health service equity and access.

### Direct health benefits

All participants commented on how participating in and attending the art activities at Fendika directly improved their health. The mechanisms include stress reduction, increased social cohesion and reduced loneliness, and increased happiness and wellbeing.

#### Stress reduction

Participants described how the music lifts feelings of depression, and they experience and witness stress relief through cultural dancing and music on stage.

“So, if I'm depressed and I find enough strength to go to Fendika by the end of it, I know I will feel better” Male1, Interview, Audience member.

“Once I repair my soul after I come here, I felt I'd leave with my soul repaired for the week or for two weeks. I'm good to go around in the world” Female1, Interview, Audience member.

#### Increased social cohesion and reduced loneliness

Participants spoke of the isolation experienced during the curfews and shelter-in-place orders during the peak of the COVID-19 pandemic and how Fendika, by opening its doors for some core artists and by streaming live music to a worldwide audience, made them feel connected. The war also created isolation—isolation from friends and family—and additional worry about their safety. Fendika was a place to find comfort and social support.

“But for a single people that lived alone, [COVID] was difficult. And fun to see a live performance - it showed that the show can go on” Male 2, Interview, Audience member.

“During the war, I'm one of the people that were personally affected …. I went to Fendika to find solace and comfort” Male1, Interview, Audience member.

“I have very deep connection with the people there [Tigray]. And whatever was happening, whenever the war was happening there, I would just imagine my friends, just imagine the family I've rented houses with from …and it was getting to me a lot. I don't think I coped with it. When I came here to release that, I came here to forget and after this I would go back to the world” Female1, Interview, Audience member.

#### Increased happiness and wellbeing

Finally, Fendika provided a place for happiness and feeling better, regardless of what was happening to them or to the country.

“Fendika is our hospital, a place for us to recover and feel better" M1, Focus Group, Staff.

“What I can say is, I'm pregnant now. I'm sick and my mind goes crazy sometimes - I'm stressed out. But when I come to Fendika and stay a while, all my systems become normal again. I'm happy I'm myself again” F1, Focus Group, Artist.

### Safe, inclusive, engaging environment

Fendika is a place that is a safe and inclusive environment for people from across socioeconomic standing, cultural identity, and other aspects of inclusion. The mechanisms by which the arts at Fendika influence the environment are through fostering cultural and historical representation, as well as civic pride and engagement.

#### Cultural and historical representation

The ethnic diversity in the country, coupled with the war, has created a lot of division. The participants universally agreed that the inclusive nature of music, dance, and other arts was a unique and vital component of Fendika as a place of cultural and historical representation—both in seeing themselves in the arts and also in understanding others through the arts.

“But if it's not my culture, watching their spirit presented that way will help you understand and appreciate more [and] brings people together” Male2, Interview, Audience member.

“And …if you are singing…from all cultures together,… they all appreciate each other's culture. [Acceptance] will change” Female, Interview, Public Health leader.

#### Civic pride and engagement

Participants shared experiences of unity, equality, and community healing from the war in Tigray at Fendika. Participants also expressed a sense of freedom to express themselves.

“And, you know, the war was taking place in Tigray and at Fendika, there were still Tigray artists performing every Friday. And in fact, Maluku sometimes would come out and say, you know, this is our lovely brother from that region that you know, he shows us love and that reminds us that regardless of our challenge we will come through” Male1, Focus Group, Artist.

“This is where the artists express themselves, their freedom” F3 Focus group, Artist.

### Social, cultural, and policy change

The arts can contribute to addressing the social and structural factors that affect health equity. The mechanisms by which are the ability of the arts to enable dialogue within or across groups, increase social cohesion, elevate underrepresented voices, and increase community capacity and resilience (21).

#### Enable dialogue within or across groups

Participants shared that the unique environment draws people from a wide spectrum of experiences and backgrounds to Fendika. In addition, the performances themselves can be provocative.

“You know, and it's a space where people with low power low status can interact with people with high status, high power in a very egalitarian way” Male1, Interview, Audience member.

“The Friday Night performances and the same thing the country was so divided with the war and two, unbelievable level that sometimes you sort of wonder if we are all humans. We, everyone was engaged in unspeakable things but Fendika never stopped performing everybody's culture. And that brings hope for the people that are pushed away” Male2, Interview, Audience member.

#### Increase social cohesion

Participants shared that Fendika provides the space for social cohesion across hierarchy and culture through their performances and an equity-minded space where all people who attend Fendika are considered equals.

“And coming here, it makes you much more united. Because, for example, she can dance everything. And she's Gurage (ethnic group). Whenever she dances she becomes Gurage for me. When she dances Oromia she becomes Oromo (ethnic group) for me. Everybody that comes here will reflect on their ethnic roots and experience their true roots” Female1, Interview, Audience member.

#### Elevating underrepresented voices

This is apparent in both the representation of artists and arts and the intentional effort to assure equity in representation. Coming from a challenging background himself, Melaku spends his energy elevating others—artists, staff, community members, and audience members.

“One of the things that is peculiar about this art gallery is it doesn't take any commissions or it doesn't engage in any kind of trade activities or commercial activities. It is simply here to contribute to the artist presenting. You don't get in other platforms and others” Male3, Focus Group, Artist.

“Melaku was a street child. Right? So somebody took him in. And, he does that to somebody else” Male2, Focus Group, Artist.

#### Increases community capacity and resilience

The philosophy and practices at Fendika enhance the community’s capacity to strive toward equity across cultures. Staff are trained in all functions of the center, increasing their individual capacity to grow themselves and their personal resilience. At a community level, the cross-cultural representation and welcoming space build the capacity for the community to recover from difficulties.

“The whole conservative system, the cultural blockade that we used to have, we just tore it apart, and it became more than a cultural space, it became a center of art” Male2, Interview, Audience member.

“During COVID time, it was hard, but [Melaku] never said he was tired. He was positive and thankful. He never stopped paying us salaries” F2, Focus group, Staff.

### Health service equity and access

Health service equity and access can be modified through the arts. Specifically, the arts increase access and engagement in health, and the arts provide a means of facilitating dialogue about difficult health issues and can be an opportunity to provide services in a more culturally responsive manner. The respondents largely did not specifically discuss health service equity and access, with the exception of the public health leader.

#### Increase access and engagement

The arts can be used to engage an emotional response from the community, thus increasing the community’s interest in the health issue and ways in which to access the care needed.

“I think music in general has a lot of benefits. And I think there is a lot of research with that. …. But a lot of people use music therapy with depression and stuff. Here [Fendika] what you get …is the energy” Female1, Interview, Audience member.

“So I believe very much that with art and something which is amusing people you can change things. You see,… take a film into a community and see what kind of conversations it sparks, what kind of new ideas they bring to the county” Female, Interview, Public Health Leader.

#### Facilitate dialogue about difficult issues

The arts can be an effective approach to changing behavior and discussing difficult health-related topics.

“I believe very much that this [the arts] is a better way of changing attitude and changing behavior than the normal behavior change of teaching knowledge” Female, Interview, Public Health leader.

#### Deliver services in a more culturally responsive manner

The use of the arts developed and delivered by people from their own communities is one important strategy for the delivery of health-related messages in a culturally responsive manner.

“*So I sent this film to the village on this Thursday, you know, for this to have an impact and the students who are graduated from here took this to show it to their communities. So this is going to change behavior, to have an impact” Female, Interview, Public Health Leader*.

## Discussion

The purpose of this study was to explore and describe the ways in which the arts can influence mental health, build social support, and create cultural unity. Fendika Cultural Center provides music, dance, visual art, and social connection through its programming for people of all ages and backgrounds for no or nominal costs. Participants universally shared the benefits of stress reduction, reducing loneliness, and social cohesion. What is perhaps unique about this center in the context of Ethiopia today is its cultural and historical representation, civic pride, and engagement through music and dance. Cross-cultural understanding and unity were experienced in the sharing of cultural dance, music, and art, thus reinforcing the values of Fendika as a place of inclusion. The cultural center increased staff, participants’, and artists’ capacity and resilience and not only elevated underrepresented voices but also intentionally drew underrepresented voices to the forefront—for example, music and dance from the Tigray region during the war. Because of cohesion and equity, Fendika supported people’s capacity for engaging in dialogue about difficult issues. The public health leader in particular noted the importance of using the arts to convey messages that reach the emotions of the person/community and change behavior.

The literature supports the benefits of arts engagement across the life course in direct and indirect ways (20). The direct benefits of engaging in the arts are improved mental and physical health (20, 26–28), support of cognitive development, and enhanced social wellbeing (20, 21, 27, 28). The mental health benefits of music and dance are not novel (29–32). Art-based activities for mental health are also well documented, although much of the research lacks rigorous design (33). For example, improvement in physical and mental health was observed in randomized older adults following a 12-week, 2-h per week art-based activity at a museum (26). Consistent with the literature, participating in the arts in a setting with other people does reduce isolation (34) and can build social cohesion (35).

Place-based arts are capable of building social cohesion and igniting a movement toward more equitable communities. Creating a space that provides discourse across groups is a step in changing the social and structural systems (36). Strategies to effectively amplify change through social cohesion include building and sharing power, connecting people across differences, assuring representation of community members with varied experiences and backgrounds, and working toward the same community-driven goals (36). Each of these strategies was observed at Fendika. Inclusive and universal Ethiopian music, dance, and art were represented across ethnic groups, including the representation of the ethnic groups engaged in armed conflict. Fendika’s mission is to “celebrate and renew Ethiopia’s rich cultural heritage. [They] welcome and nurture all creative souls; through the exchange of music, dance, art, and poetry, we meditate on peace and humanity’s one-ness” (22). Fendika intentionally sought representation to build unity and equity.

From a public health institutional perspective, there is compelling evidence to show the potential for health behavior change with the use of the arts (37) and that the arts have been effective for health behavior change. For example, “Telanovelas” have been used across communities and topics of health behavior change. A randomized control trial was conducted in which Latina participants viewed a video versus a pamphlet to reduce stigma and increase mental health literacy. The video intervention condition experienced significantly higher health literacy than the comparison condition (38). In the current study, the public health professional described using a video to improve health outcomes in local communities by engaging an emotional response through the arts mechanism. While this is of secondary importance for this study, the complex health and social conditions in Ethiopia offer an opportunity for the public health system to build on existing evidence and use the arts to enhance community mental health, build social cohesion, and support cross-cultural understanding and acceptance.

There are several limitations to this study. Fendika Cultural Center is one example, and it is unknown whether the environment of Fendika can be replicated or generalizable. Given the use of purposeful and word-of-mouth recruitment, self-selection bias may have been introduced, as participants may have joined the study because of their support for Fendika, thus not representing a range of experiences. The analysis was led by a faculty member with no prior relationship with Fendika, with the intent to limit subjective bias during the analysis. The selection of an *a priori* evidence-based framework and deductive analysis was another strategy employed to reduce subjective bias. While the results cannot be generalized to all of Ethiopia, the findings are consistent with existing literature and the value of the arts in supporting mental health and wellbeing.

## Conclusion

This and other studies show the importance of the role of the arts in community mental health, social support, and creating cultural unity. Additional research is needed, including a broader representation of participants of Fendika and from the surrounding community. Both qualitative and quantitative research studies are needed to further understand the mechanisms of the different modes of ‘art’ on mental health and wellbeing in this context and if the positive impact is sustained over time. For example, do the feelings of cohesion and cultural understanding remain when engaging with multiple ethnic groups in the community? It is also important to assess the role of the arts in general across the country. Addis Ababa is a large, urban, and international center. The ethnic community facing the most conflict and strain was likely not represented here. Further research should apply more rigorous study designs and assess the replication of effective models into new communities. Regardless, the arts appear to have the potential to improve the mental health crisis and intervene in the complex, divisive, and toxic social and political environments experienced by so many communities.

## Data availability statement

The raw data supporting the conclusions of this article will be made available by the authors, without undue reservation.

## Ethics statement

The studies involving humans were approved by Saint Catherine University IRB approved this research. The studies were conducted in accordance with the local legislation and institutional requirements. The participants provided their written informed consent to participate in this study.

## Author contributions

MH: Formal analysis, Methodology, Writing – original draft, Writing – review & editing. MB: Data curation, Writing – review & editing, Supervision, Validation. HW: Data curation, Writing – review & editing, Conceptualization, Methodology.

## Footnotes

^1^ https://fendika.org/about
